# Catalytically inactive carbonic anhydrase‐related proteins enhance transport of lactate by MCT1

**DOI:** 10.1002/2211-5463.12647

**Published:** 2019-06-11

**Authors:** Ashok Aspatwar, Martti E. E. Tolvanen, Hans‐Peter Schneider, Holger M. Becker, Susanna Narkilahti, Seppo Parkkila, Joachim W. Deitmer

**Affiliations:** ^1^ Faculty of Medicine and Health Technology Tampere University Finland; ^2^ Department of Future Technologies University of Turku Finland; ^3^ Division of General Zoology FB Biologie TU Kaiserslautern Germany; ^4^ Present address: Department of Physiological Chemistry University of Veterinary Medicine Hannover Germany; ^5^ Present address: NeuroGroup BioMediTech Tampere Finland; ^6^ Present address: Fimlab Laboratories Ltd. Tampere University Hospital Finland

**Keywords:** carbonic anhydrase‐related protein, lactic acid, MCT1, membrane transport, transporter

## Abstract

Carbonic anhydrases (CA) catalyze the reversible hydration of CO_2_ to protons and bicarbonate and thereby play a fundamental role in the epithelial acid/base transport mechanisms serving fluid secretion and absorption for whole‐body acid/base regulation. The three carbonic anhydrase‐related proteins (CARPs) VIII, X, and XI, however, are catalytically inactive. Previous work has shown that some CA isoforms noncatalytically enhance lactate transport through various monocarboxylate transporters (MCT). Therefore, we examined whether the catalytically inactive CARPs play a role in lactate transport. Here, we report that CARP VIII, X, and XI enhance transport activity of the MCT MCT1 when coexpressed in *Xenopus* oocytes, as evidenced by the rate of rise in intracellular H+ concentration detected using ion‐sensitive microelectrodes. Based on previous studies, we suggest that CARPs may function as a ‘proton antenna’ for MCT1, to drive proton‐coupled lactate transport across the cell membrane.

**Abbreviations**
CA: carbonic anhydrase
CARP: carbonic anhydrase‐related protein
MCT: monocarboxylate transporter
qPCR: quantitative PCR

The monocarboxylate transporter (MCT) family, also known as SLC16, consists of 14 isoforms 1. Among them, MCT1 is ubiquitous and predominantly expressed in the tissues that require large amounts of energy, like brain and muscle 2. In the brain, the export of lactate by MCT1 is required to provide lactate for the energy metabolism of neurons from astrocytes in the glia‐neuron lactate shuttle, in which MCT1 exports lactate from the astrocytes, to be taken up by neurons through the high‐affinity MCT2 3, 4. This is significant for neuroprotection, especially in glucose‐deprived conditions 5, 6. In addition to the brain, lactate has also been reported as preferred fuel under stress/strain conditions in heart and skeletal muscle, and perhaps lactate also serves as a signaling molecule in such conditions (reviewed in Ref 7). Already moderate physical activity doubled the contribution of lactate for total cardiac energy production in healthy subjects 8, while heavy exercise (at 200 W) increased lactate uptake by a factor of four, with a 60% contribution to cardiac energy production 9, 10. Studies on rats demonstrated that increased blood lactate levels can have positive effects on heart function during a septic or hemorrhagic shock 11, 12.

In mammals, the major role of alpha‐carbonic anhydrases (α‐CAs) is to catalyze the reversible hydration of CO_2_ to ${\text{HCO}}_{3}^{-}$ and H^+^ to regulate pH in a variety of tissues 13. The involvement of CAs in epithelial transport of ions and fluids, in particular in kidneys, also contributes in regulating the whole‐body acid/base balance. Apart from pH modulation, the α‐CAs also associate with transporter proteins forming transport metabolons, which facilitate the transport of various anions across the membrane 14. This may occur through equilibration of cotransported ${\text{HCO}}_{3}^{-}$ or H^+^ species. Transport activity of MCTs is facilitated by various CA isoforms via a mechanism that is independent from the enzymes’ catalytic activities 15, 16, 17, 18, 19, 20, 21, 22, 23, 24, 25, 26, 27. Intracellular CAII, but not CAI and CAIII, facilitates transport activity of MCT1 and MCT4, when heterologously expressed in *Xenopus* oocytes 15, 16, 17, 18, 19, 20. CAII‐mediated facilitation of MCT1/4 activity is independent from CAII catalytic function, but requires direct binding of the enzyme to a cluster of three glutamic acid residues in the transporters’ C‐terminal tail 19, 23. Transport activity of MCT2, which lacks a CAII binding site, is not facilitated by CAII 18. However, introduction of three glutamic acid residues into the MCT2 C‐terminal tail allowed binding of CAII to the transporter and enabled CAII‐mediated facilitation of MCT2 transport activity 23. Binding of CAII to the transporter is mediated by CAII‐His64 22. Interestingly, His64 resembles the central residue of the CAII intramolecular proton shuttle 28. It has been suggested that CAII serves as a ‘proton antenna’ for MCTs, which mediates the rapid exchange of protons between transporter pore and surrounding protonatable residues 17, 22, 29. In CAII, proton shuttling between enzyme and transporter seems to be mediated by CAII‐Glu69 and CAII‐Asp72, which form a surface proton antenna on the enzyme, while CAII‐His64 mediates binding to the transporter, but no proton exchange 22. CAII does not only facilitate MCT transport activity in *Xenopus* oocytes, but can also drive lactate flux in astrocytes 19 and cancer cells 22 by noncatalytic function. Transport activity of MCT1, MCT2, and MCT4 was further shown to be enhanced by the extracellular CA isoforms CAIV and CAIX 18, 20, 21, 26, 27. CAIV‐mediated facilitation of MCT transport activity, as expressed in *Xenopus* oocytes, is independent from the enzyme's catalytic activity, but requires direct binding of CAIV‐His88 (the analogue residue to CAII‐His64) to the Ig1 domain of the MCT chaperons CD147 (MCT1, MCT4) and GP70 (MCT2), respectively 18, 27. Facilitation of MCT‐mediated lactate flux by CAIX was demonstrated in *Xenopus* oocytes and hypoxic breast cancer cells, where the CAIX‐induced increase in lactate transport capacity supports cell proliferation under hypoxia 21, 26. Proton shuttling between MCTs and CAIX is partially mediated by the CAIX proteoglycan‐like domain that is rich in acid residues and might serve as proton antenna for the transporter 26.

In the present study, we have investigated the possible role for carbonic anhydrase‐related proteins (CARPs) VIII, X, and XI in the transport of lactate in association with MCT1. CARPs VIII, X, and XI are catalytically inactive proteins and are predominantly expressed in the human brain 30, 31. Because of the lack of enzymatic activity, the CARPs are assumed to function through interaction with other proteins. 32.

In case of CARP VIII, there is a known interaction with inositol 1,4,5‐trisphosphate receptor type 1 to modulate Ca^2+^ release from endoplasmic reticulum into cytoplasm 33. Several CA8 loss‐of‐function‐associated phenotypes of poor motor coordination have been reported in human, mouse, and zebrafish 34, 35, 36, 37, consistent with CARP VIII being predominantly expressed in the cerebellum.

Downregulation of CARP Xa or CARP Xb in zebrafish leads to defects in the development of brain and an ataxic swim pattern, reminiscent of the effects of CARP VIII knockdown 38. Recent studies in mouse brain by Sterky *et al*. 39 have shown that CARP X and CARP XI dimerize with neurexin‐1 through a membrane‐proximal disulfide bond and that the complex formation enhances the surface expression of neurexin‐1 39. In this study, we wanted to see whether CARPs would have effects on proton‐coupled lactate transport similar to the noncatalytic enhancement by other CAs 20. We have coexpressed MCT1 with the CA isoforms VIII, X, and XI in *Xenopus* oocytes and determined MCT1 and CA activity by measuring the rate of change in intracellular H^+^ concentration (ΔH^+^/Δ*t*) with ion‐sensitive microelectrodes. Our results show that all three CARPs functionally interact with the MCT1 and enhance the transport activity of MCT1.

## Materials and methods

### Generation of hCA8 gene from human neuronal cells

Total RNA was isolated from 8 + 2‐week‐old human neuronal cells using Qiagen kit for RNA isolation for cultured cells (Qiagen, Hilden, Germany). Total RNA was isolated from 30 mg sample using the RNeasy® Mini kit (Qiagen) by following the manufacturer's instructions. The concentration and purity of total RNA were determined using a Nanodrop Spectrophotometer at 260 and 280 nm. Reverse transcriptase PCR was performed using 0.1–5 μg of total RNA to synthesize the first‐strand cDNA using First Strand cDNA Synthesis kit (High‐Capacity cDNA Reverse Transcription Kits; Applied Biosystems, Foster City, CA, USA) with random primers and M‐MuLV reverse transcriptase according to the protocol recommended by the manufacturer.

### Cloning of human CARP genes in pGEM‐He‐Juel vector

The human *CA10* and *CA11* obtained from IMAGE (MGC Geneservice Ltd, Cambridge, UK) and human *CA8* gene were generated by RT/PCR from pluripotent human neuronal cells as described above and were inserted into pGEM‐He‐Juel using the primers given in Table 1. PCR amplification of all three human CARP genes was carried out using the forward and reverse primers containing the restriction sites for appropriate restriction enzymes (Table 1) using the PCR conditions: denaturation at 98 °C for 2 min, 35 cycles of denaturation at 98 °C for 10 s, annealing at 55 °C for 30 s, extension at 72 °C for 1 min, and extension at 72 °C for 10 min.

**Table 1:** Primers used in the experiments for cloning and qPCR analysis

Gene name	Name of the primer	Primers for cloning	Primers for qPCR
hCA8	hCA8BamHI_F	cgcggatccatggcggacctgagcttcat	tgctttaatcccaacaccttattacc
	hCA8EcoRI_R	ccggaattcctactgaaatgcagctctaatgac	tggcattgtaagagatccctcat
hCA10	hCA10 BamHI_F	cgcggatccatggaaatagtctgggaggtgct	gttggtggacatataaggaggttgt
	hCA10EcoRI _R	ccggaattcctacttgaggagccattcatt	ttaccaagccccaaaaggaa
hCA11	hCA11BamHI _F	cgcggatccatgggggctgcagctcgtctg	tccgctcaggctgagtatga
	hCA11EcoRI _R	ccggaattctcagcgaccatgggggacacc	gaaacatggcgccctgtatt

The amplified product of the CARP genes and the plasmid vector pGEM‐He‐Juel were digested with the suitable restriction enzymes. The digested products were purified by MinElute kit (Qiagen) and then ligated by the T4 ligation system (Promega, Madison, WI, USA) and cloned in One Shot® TOP10 competent cells by taking 1 μL of the plasmid plus 25 μL of competent cells and incubated on ice for 30 min. The cells were heat‐shocked at 42 °C for 30 s and transferred to the ice for 2 min. 125 μL of SOC medium was added to each tube and kept at 37 °C in a shaker at 225 r.p.m. for 1 h. 20 μL of the cells was spread on Luria/Bertani (LB) agar plates and incubated at 37 °C for 16 h. The bacterial colonies were screened by colony PCR for the presence of the correct insert. The DNA sequencing of four different clones for each CARP gene was carried out. The sequences thus obtained were aligned with ClustalW 40 and compared with cDNAs from the databases.

### Heterologous protein expression in *Xenopus* oocytes

The procedure of heterologous protein expression in *Xenopus* oocytes has been described in detail previously 41, 42. In brief, cDNA coding for human the CA isoforms VIII, X, and XI, and rat MCT1, respectively, cloned into pGEM‐He‐Juel, was transcribed *in vitro* using T7 RNA‐Polymerase (mMessage mMachine, Ambion Inc., Austin, TX, USA). Frogs were purchased from the Radboud University, Nijmegen, the Netherlands. Segments of ovarian lobules were surgically removed under sterile conditions from *Xenopus laevis* females which were anesthetized with ethyl 3‐aminobenzoate methanesulfonate (Tricaine, MS‐222; Sigma‐Aldrich, Schnelldorf, Germany), and rendered hypothermic. The procedure was approved by the Landesuntersuchungsamt Rheinland‐Pfalz, Koblenz (23 177‐07/A07‐2‐003 §6). Oocytes were singularized by treatment with collagenase (Collagenase A; Roche, Mannheim, Germany) in Ca^2+^‐free oocyte saline (pH 7.8) for up to 2 h at 28 °C. Singularized oocytes were incubated at 18 °C overnight in Ca^2+^‐containing oocyte saline (pH 7.8) to recover. Oocytes of the developmental stages V and VI were injected with 3 ng of cRNA coding for MCT1, either together with 15 ng of cRNA coding for CA VIII, CA X, and CA XI, respectively, or alone. Measurements were carried out 3–6 days after injection of cRNA.

The oocyte saline had the following composition (in mm): NaCl, 82.5; KCl, 2.5; CaCl_2_, 1; MgCl_2_, 1; Na_2_HPO_4_, 1; 4‐(2‐hydroxyethyl)‐1‐piperazineethanesulfonic acid (HEPES), 5; titrated with NaOH to the desired pH. In lactate‐ and CO_2_/${\text{HCO}}_{3}^{-}$‐containing saline, NaCl was substituted by equimolar amounts of Na‐L‐lactate or NaHCO_3_.

### Measurement of intracellular H^+^ concentration in *Xenopus* oocytes

Changes in [H^+^]_i_ were determined with ion‐sensitive microelectrodes under voltage‐clamp conditions, using double‐barreled microelectrodes. Manufacture and application of the electrodes have been described previously 41, 42. In brief, two borosilicate glass capillaries with a diameter of 1.0 and 1.5 mm were twisted together and pulled to a micropipette. The tip of the ion‐sensitive barrel was filled with 5% tri‐*N*‐butylchlorsilane in 99.9% pure carbon tetrachloride and baked for 4.5 min at 450 °C on a hot plate. A drop of H^+^‐sensitive cocktail (95291, Sigma‐Aldrich, Schnelldorf, Germany) was backfilled into the silanized tip, and the barrel was filled up with 0.1 m Na‐citrate, pH 6.0. The reference barrel was filled with 3 m KCl. Calibration of the electrodes was carried out in oocyte salines with a pH of 7.0 and 6.4. To detect optimal H^+^ changes, the electrode was located near the inner surface of the plasma membrane, as described previously 43. Oocytes were constantly clamped to a holding potential of −40 mV during the whole course of the experiment with an additional microelectrode, filled with 3 m KCl which was connected to an Axoclamp 2B amplifier (Axon Instruments, Foster City, CA, USA). All experiments were carried out at room temperature (22–25 °C). The measurements were recorded with a custom‐made software tool, based on the program LabView (National Instruments Germany GmbH, München, Germany). For determination of Δ[H^+^]_i_/Δ*t*, the initial slope of the H^+^ signal was determined by linear regression using originpro 8.6 (OriginLab Corporation, Northampton, MA, USA) as previously described 41.

### Real‐time quantitative PCR of human CARP and MCT1 genes from *Xenopus* oocytes

Real‐time quantitative PCR (qPCR) primers were designed based on the transcript sequences taken from Ensembl (www.ensembl.org; ENST00000317995, ENST00000084798, ENST00000285273, and ENST00000369626 for *CA8*,* CA10*,* CA11*, and *SLC16A1*, respectively), using the program Primer Express® Software v2.0 (Applied Biosystems). Real‐time qPCR was performed using the SYBR Green PCR Master Mix Kit in an ABI PRISM 7000 Detection System™ according to the manufacturer's instructions (Applied Biosystems). The PCR conditions consisted of an initial denaturation step at 95 °C for 10 min followed by 40 cycles at 95 °C for 15 s (denaturation) and 60 °C for 1 min (elongation). The data were analyzed using the ABI PRISM 7000 SDS™ software (Applied Biosystems). Every PCR was performed in a total reaction volume of 15 μL containing 2 μL of first‐strand cDNA (20 ng cDNA), 1 × Power SYBR green PCR Master Mix™ (Applied Biosystems), and 0.5 μm of each primer. The final results expressed as the N‐fold relative difference (ratio) in gene expression between the studied samples. The relative expression values were calculated according to the equation of Pfaffl with appropriate modification 44.

## Results

### CARPs enhance transport activity of MCT1 in *Xenopus* oocytes

To investigate whether CARPs can enhance the transport activity of MCT1, the rate of rise in intracellular H^+^ concentration (Δ[H^+^]_i_/Δ*t*) was determined in oocytes, expressing MCT1 alone or coexpressing MCT1 and CARP VIII, X, or XI, respectively, during application of 3 or 10 mm lactate (Fig. 1A). Since lactate is transported by MCT1 with H^+^ in a 1 : 1 stoichiometry, Δ[H^+^]_i_/Δ*t* can be used as a direct measure for MCT transport activity. Coexpression of any of the three CARPs resulted in a significant increase in Δ[H^+^]_i_/Δ*t* by 54–86%, indicating that the CARPs VIII, X, and XI indeed enhance MCT1 transport activity (Fig. 1B). In H_2_O‐injected control oocytes, lactate application induced no change in [H^+^]_i_, confirming that the lactate‐induced changes in intracellular H^+^ concentration in MCT1‐expressing oocytes are mediated by MCT1 transport activity.

**Figure 1:** Catalytically inactive CARP VIII, X, and XI facilitate MCT1 transport activity. (A) Original recordings of intracellular H^+^ concentration in oocytes expressing MCT1 (black trace), or coexpressing MCT1 + CA8 (green trace), MCT1 + CA10 (red trace), and MCT1 + CA11 (blue trace), respectively, during application of 3 and 10 mm lactate. (B) Rate of changes in intracellular H^+^ concentration (Δ[H^+^]_i_/Δ*t*) as induced by application of 3 and 10 mm lactate, respectively, in oocytes expressing MCT1 (black), or coexpressing MCT1 + CA8 (green), MCT1 + CA10 (red), and MCT1 + CA11 (blue). Left‐hand bars in each pair correspond to 3 mm lactate and right‐hand bars to 10 mm lactate, as indicated in the green bars. (C) Original recordings of intracellular H^+^ concentration in oocytes expressing MCT1 (black trace), or coexpressing MCT1 + CA8 (green trace), MCT1 + CA10 (red trace), and MCT1 + CA11 (blue trace), respectively, during application of 5% CO_2_/10 mm ${\text{HCO}}_{3}^{-}$. (D) Rate of changes in intracellular H^+^ concentration (Δ[H^+^]_i_/Δ*t*) as induced by application of 5% CO_2_/10 mm ${\text{HCO}}_{3}^{-}$, respectively, in oocytes expressing MCT1 (black), or coexpressing MCT1 + CA8 (green), MCT1 + CA10 (red), and MCT1 + CA11 (blue). The numbers above the bars refer to number of experiments *n*. All values are depicted as mean + SEM. *Significance level of *P* ≤ 0.05, **significance level of *P* ≤ 0.01; n.s., no significance (Student's *t*‐test, as compared to oocytes with MCT1 expressed alone). (E) Original recording of intracellular H^+^ concentration in a H_2_O‐injected control oocyte during application of 3 and 10 mm lactate and 5% CO_2_/10 mm ${\text{HCO}}_{3}^{-}$.

Potential catalytic activity of CARPs was checked by measuring Δ[H^+^]_i_/Δ*t* during application of 5% CO_2_/10 mm ${\text{HCO}}_{3}^{-}$ in oocytes, expressing MCT1 alone or coexpressing MCT1 and CARP VIII, X, or XI, respectively (Fig. 1C). Application of CO_2_/${\text{HCO}}_{3}^{-}$ evoked an increase in [H^+^]_i_, the rate of which did not significantly differ between the four types of oocytes (Fig. 1D). The values are also similar to those recorded in H_2_O‐injected oocytes (Fig. 1E) 45. These results confirm that none of the three CARPs exhibits CA catalytic activity.

Levels of the human genes added by cRNA injections were measured by RT–qPCR. Figure 2 shows that the expected genes were observed at similar levels. Panels A to C show the levels of CA8, CA10, and CA11 sequences, respectively, and Panel D shows that of MCT1. The level of each gene was at RT–qPCR background levels when the corresponding cRNA was not injected.

**Figure 2:** Presence of CARP genes in injected *Xenopus* oocytes measured by RT–qPCR. Labels under the columns indicate the injected genes, native meaning not injected with any human gene. Measured transcripts of A, *CA8*; B, *CA10*; C, *CA11*; and D, *SLC16A1* (*MCT1*). The bar graphs are the average values of three replicates (*n* = 10 in each group), and the error bars indicate standard deviation (SD).

## Discussion

We have observed a clear enhancement of transport activity of MCT1 by coexpression of MCT1 with any of the human CARPs (VIII, X, and XI). These proteins are devoid of CA enzymatic activity due to missing histidines in the active site, so the assistance provided by CARPs is definitely noncatalytic. Previous studies have shown that facilitation of MCT1 by intracellular CA II is independent of the CA catalytic activity, but requires the enzymes’ intramolecular proton shuttle with the histidine at position 64 and the two acidic residues Glu69 and Asp72, which could function as surface proton collectors for the enzyme 17, 22. From this, it was concluded that CA II could function as a ‘proton antenna’ for the transporter, which can rapidly move H^+^ between the transporter pore and surrounding protonatable residues. The need for such an antenna derives from the finding that H^+^ cotransporters such as MCTs, substrate of which is available only at very low concentrations, extract H^+^ from the surrounding area at rates well above the capacity for simple diffusion to replenish their immediate vicinity. Therefore, the transporter must exchange H^+^ with protonatable sites at the plasma membrane, which could function as a ‘proton‐harvesting antenna’ for the transporter 29. Intracellular CA II, when directly bound to MCT1 or MCT4, can move protons between the transporter pore and surrounding protonatable residues at the cytosolic face of the plasma membrane, which dissipates local proton microdomains and facilitates H^+^/lactate cotransport 15, 17. We assume that CARP VIII, X, and XI could also function as ‘proton antenna’ for MCT1 to facilitate proton‐coupled transport, in a similar way as is suggested for other CAs. Even if the shuttling‐mediating residues Glu69 and Asp72 of CA II 22 are not conserved in any of the CARPs, there are other acidic residues on their surfaces near the ‘active‐site cavity’ which could work in the same function. A more detailed study is ongoing in our laboratories. Interestingly, the intramolecular proton shuttle, His 64, is conserved among all three CARPs 46. Therefore, it appears plausible that the MCT1 C‐terminal tail might bind in the cavity in the same way as noted for CA II 22.

Carbonic anhydrase‐related proteins VIII is an intracellular protein, whereas CARPs X and XI are secretory 38. Since all three isoforms enhance MCT1 transport activity, it can be assumed that CARPs can interact with MCT1 both on the intracellular and on the extracellular site. Indeed, the previous experiments have shown that also the extracellular enzymes CA IV and CA IX can facilitate the MCT transport activity 18, 20, 21. Intracellular CA II has been shown to bind to an acidic cluster in the C‐terminal tail of MCT1 and MCT4, respectively 19, 23, while extracellular CA IV and CA IX might interact with the transporter via its chaperon CD147 20, 21. From this, it can be assumed that CARP VIII interacts with MCT1 by binding to the transporter's C‐terminal tail, while CARP X and CARP XI would interact with the transporters chaperon CD147 on the extracellular site.

Emerging data indicate that the CARP proteins interact with several proteins. We are currently studying complex‐forming partners of CARP X in human pluripotent stem cell ‐derived neurons by mass spectrometry proteomics, and the preliminary results implicate many novel binding partners (which will be reported later), some of which may be disulfide‐bonded. We propose that the secretory CARPs (X and XI) have a general tendency to block unpaired cysteines and thus form many types of disulfide complexes with other proteins that are being synthesized, even for other proteins than the documented case of neurexin‐1 39. The disulfide bonding is mediated by the C‐terminal extension in CARPs X and XI, after the CA domain 38, 39. Therefore, the CA domain should be mainly unchanged after binding and completely accessible for interactions even when CARP X and CARP XI are parts in covalent complexes.

## Conflict of interest

The authors declare no conflict of interest.

## Author contributions

AA, MT, HMB, SP, and JWB designed the study; AA, HPS, HWB, and SN performed experiments; AA, MT, HPS, HWB, JWB, and SN analyzed and interpreted the data; AA, MT, HWB, JWB, SN, and SP wrote the paper; all authors revised the manuscript in various stages; and HMB, JWB, and SP provided resources for the study.
